The article "CX3CL1 Derived from Bone Marrow Mesenchymal Stem Cells Inhibits Aβ1-42-Induced SH-SY5Y Cell Pathological Damage through TXNIP/NLRP3 Signaling Pathway" was retracted in 2023. Reasons: unreliable results or conclusions; concerns about the data; concerns about the peer review; concerns about the citations.

# CX3CL1 Derived from Bone Marrow Mesenchymal Stem Cells Inhibits A*β*_1-42_-Induced SH-SY5Y Cell Pathological Damage through TXNIP/NLRP3 Signaling Pathway

**DOI:** 10.1155/2022/1949344

**Published:** 2022-09-08

**Authors:** Chuan Guo, Qinxuan Li, Jiujia Xiao, Xuhui Zhou, Meichen Tian, Lei Xie, Xun Xia

**Affiliations:** ^1^Chengdu Medical College, Chengdu Sichuan 610500, China; ^2^Department of Critical Care Medicine, The First Affiliated Hospital of Chengdu Medical College, Chengdu Sichuan 610500, China

## Abstract

Alzheimer's disease (AD) is the most commonly seen neurodegenerative brain disorder. The paracrine effects of mesenchymal stem cells (MSCs) signify to trigger immunomodulation and neural regeneration. However, the role and mechanism of bone marrow MSC- (BMSC-) derived CX3CL1 in AD remains elusive. In this study, A*β*_1-42_-intervened SH-SY5Y cells were used for AD cell model construction. pcDNA-ligated CX3CL1 overexpression plasmids were transfected into BMSCs. The levels of soluble and membrane-bound CX3CL1 were detected by ELISA and Western blotting (WB), respectively. The growth, apoptosis, and pathology of AD model cells were evaluated by CCK-8, flow cytometry, immunofluorescence, morphology observation, biochemical examination, and WB. It was found that A*β*_1-42_ significantly reduced CX3CL1 expression either in soluble or membrane-bound form, cell viability, relative protein expression of synaptic markers, SOD, CAT, and GSH-Px contents, as well as Trx protein expression; in addition, it enhanced the apoptosis rate, the relative expression of cleaved caspase-3, A*β*, tau, p-Tau, Iba1, MDA, TXNIP, and NLRP3 in SH-SY5Y cells; however, the above effects were prominently reversed by the coculture of BMSCs. Moreover, overexpression of CX3CL1 in BMSCs observably strengthened the corresponding tendency caused by BMSCs. In conclusion, through the TXNIP/NLRP3 pathway, CX3CL1 derived from BMSCs inhibited pathological damage in A*β*_1-42_-induced SH-SY5Y.

## 1. Introduction

As a progressive neurodegenerative brain disease, Alzheimer's disease (AD) is acknowledged to be the prime reason for dementia [1]. It is also the sixth main cause of death, with an estimate of about 75.6 million and 135.5 million sufferers worldwide as well as $2.54 trillion and $9.12 trillion costs by 2030 and 2050, respectively [2, 3]. AD is pathologically featured by the accumulation of aggregated *β*-amyloid (A*β*) plaques and neurofibrillary tangles (NFTs) that consist of hyperphosphorylated Tau proteins [4]. Thus, therapies targeting A*β* and antitau agents have attracted extensive attention [5]. However, the benefits and side effects of even the promising anti-A*β* drug, aducanumab, still need further investigations [6, 7]. Besides, antitau vaccine (AADvac1) and monoclonal antitau antibodies, including gosuranemab, tilavonemab, zagotenemab, and semorinemab, have only arrived phase II at present [5]. Even several clinical drugs, such as galantamine, memantine, donepezil, and rivastigmine, only show modest benefits to symptomatic patients with AD [8]. Therefore, potential mechanisms and therapeutic strategies for AD necessitate more attention.

The article "CX3CL1 Derived from Bone Marrow Mesenchymal Stem Cells Inhibits Aβ1-42-Induced SH-SY5Y Cell Pathological Damage through TXNIP/NLRP3 Signaling Pathway" was retracted in 2023. Reasons: unreliable results or conclusions; concerns about the data; concerns about the peer review; concerns about the citations.

As a type of pluripotent progenitor cells that can be separated from various tissues like bone marrow, fatty tissue, and umbilical cord blood, mesenchymal stem cells (MSCs) have the advantages of high proliferation and easy manipulation [9]. MSCs possess multifaceted functions, such as differentiating into glial and neuronal cells, secreting growth factor and anti-inflammatory cytokines, modulating immune cells, and stimulating endogenous repair mechanisms [10, 11], making them a novel and promising therapy for AD [12]. Bone marrow MSCs (BMSCs) are shown to alleviate cognitive decline of AD model rats [13]. Bae et al. [14] also presented that BMSCs decreased A*β* deposits and ameliorated synaptic transmission in AD mice models. Kim et al. [15] demonstrated the feasibility of AD treatment by human umbilical cord blood MSCs (hUC-MSCs) via stereotactic brain injection in a phase 1 clinical trial. Lee et al. [16] displayed that BMSCs induced the reduction of A*β* deposits and promoted microglia activation in AD mice models. Thus, MSCs are a potential and effective approach for the treatment of AD.

It has been demonstrated that the clinical efficacy of MSCs may be related to their paracrine effects on other effector cells [17]. It was found in vitro and in vivo that the suppression of BMSC-derived exosomal miR-1231 plays a role in restricting the characteristics of pancreatic cancer [18]. While supporting acute myeloid leukemia bioenergetics, BMSCs can also enhance antioxidant defense and escape from chemotherapy [19]. Meanwhile, MSCs can modulate the activation of retinal microglia by chemokine CX3CL1 signaling [20]. Moreover, CX3CL1-expressing MSCs played neuroprotective and immunomodulatory roles in the retinal degeneration rat model [21]. Also known as fractalkine, chemokine CX3CL1 is the one and only member of the CX3C family that binds to its just receptor, CX3CR1, which is expressed on the surface of microglia [22, 23]. CX3CL1 is mainly distributed in neurons within the central nervous system (CNS) [24]. Thus, there is a signaling network formed by the binding of CX3CL1 and CX3CR1 between neurons and microglia in the physiological CNS [25, 26]. There are two forms of CX3CL1 in CNS, namely, membrane-bound and soluble CX3CL1. Therein, membrane-bound CX3CL1 can be protease-cleaved to produce soluble CX3CL1 [27, 28]. Reportedly, CX3CL1 is neuroprotective via the reduced microglial generation of inflammatory factors [24]. However, the role of CX3CL1 derived from MSCs in the development and progression of AD remains elusive.

The article "CX3CL1 Derived from Bone Marrow Mesenchymal Stem Cells Inhibits Aβ1-42-Induced SH-SY5Y Cell Pathological Damage through TXNIP/NLRP3 Signaling Pathway" was retracted in 2023. Reasons: unreliable results or conclusions; concerns about the data; concerns about the peer review; concerns about the citations.

Accordingly, the motivation and novelty of this work is to clarify the role played by BMSC-derived CX3CL1 and the underlying mechanisms via A*β*_1-42_-induced SH-SY5Y cell model establishment. BMSC-derived CX3CL1 inhibited A*β*_1-42_-induced SH-SY5Y cell pathological damage via the TXNIP/NLRP3 axis.

## 2. Materials and Methods

### 2.1. Cells and Cultivation

BMSCs and the human neuroblastoma SH-SY5Y cells, supplied by Cyagen Biosciences Inc. (Guangzhou, China) and Procell (CL-0208, Wuhan, China), respectively, were cultivated under the conditions of 5% carbon dioxide (CO_2_) at 37°C in a medium comprising Dulbecco's modified Eagle's medium (DMEM; Invitrogen, Carlsbad, CA, USA) as well as 10% fetal bovine serum (FBS; Gibco, Rockville, MD, USA) and 1% streptomycin-penicillin (Solarbio, Beijing, China).

### 2.2. BMSC Transfection

BMSCs were cultivated (5% CO_2_, 37°C) after being seeded at 1 × 10^4^ cells/cm^2^ into the wells of 6-well plates. When the cell confluency reached 80%, 50 ng pcDNA-ligated CX3CL1 overexpression plasmid (CX3CL1-ov) and its corresponding empty vector plasmid (NC-ov) supplied by RiboBio (Guangdong, China) were added for transfection following Lipofectamine® 3000 (Invitrogen; Thermo Fisher Scientific, Waltham, MA, USA) recommendations. The media were replaced with DMEM after 6 h of transfection, and BMSCs were then cultured for 72 h for further assays.

### 2.3. Experimental Groups and Treatment

SH-SY5Y cells were grouped as follows: control, A*β*, A*β*+MSC, A*β*+MSC-NC-ov, and A*β*+MSC-CX3CL1-ov. An AD cell model was built via treating SH-SY5Y with 20 *μ*M A*β*_1-42_ [29], while the control group was administrated with phosphate buffer saline (PBS) with an equal amount. Moreover, SH-SY5Y cells in A*β*+MSC, A*β*+MSC-NC-ov, and A*β*+MSC-CX3CL1-ov groups were coincubated with BMSCs, BMSCs transfected with NC-ov, and BMSCs transfected with CX3CL1-ov, respectively. The observation of cell morphology and axon growth was performed with a microscope (Olympus, Tokyo, Japan). After 48 h of coculture, SH-SY5Y cells at the plate bottom were trypsinized and prepared for the following assays.

### 2.4. Enzyme-Linked Immunosorbent Assay (ELISA)

Soluble CX3CL1 concentration in cell culture supernatant, generated after 18 hours of incubation in the complete medium, was detected by commercial human fractalkine/CX3CL1 ELISA kit (ab100522, Abcam, Cambridge, UK) based on the operating instructions.

The article "CX3CL1 Derived from Bone Marrow Mesenchymal Stem Cells Inhibits Aβ1-42-Induced SH-SY5Y Cell Pathological Damage through TXNIP/NLRP3 Signaling Pathway" was retracted in 2023. Reasons: unreliable results or conclusions; concerns about the data; concerns about the peer review; concerns about the citations.

### 2.5. Western Blotting Analysis

SH-SY5Y cells after three PBS rinses were immersed in a RIPA lysis buffer (Boster, Wuhan, China) to obtain the total proteins. Following isolation by 10% SDS-PAGE, the protein samples were processed for electrical transfer onto PVDF membranes (EMD Millipore, Billerica, MA, USA) that were then sealed at an ambient temperature in bovine serum albumin (BSA; 3%) for 60 minutes and subsequently cultivated at 4°C with the following *Ι* antibodies all ordered from Abcam overnight: CX3CL1 (1 : 1000, ab25088), cleaved caspase-3 (1 : 500, ab2302), A*β* (1 : 1000, ab11132), tau (1 : 10000, ab76128), phosphorylated tau (p-Tau) (1 : 50000, ab109390), SNAP25 (1 : 1000, ab41455), Synapsin1 (1 : 1000, ab64581), PSD95 (1 : 1000, ab18258), TXNIP (1 : 2000, ab188865), Trx (1 : 1000, ab26320), and NLRP3 (1 : 1000, ab263899). At an ambient temperature, they were cultured with the corresponding II antibody for 60 minutes after triple PBS washes. Protein expressions were analyzed relative to *β*-actin. Band visualization was made with an ECL kit (EMD Millipore) based on the operating manual. Image-ProPlus (Media Cybernetics, Inc., Rockville, MD, USA) determined the gray value.

### 2.6. Cell Counting Kit-8 Assay

After each group of SH-SY5Y cells were planted into 96-well plates at 1 × 10^5^/well for overnight cultivation under the conditions of 5% CO_2_ and 37°C, the cell proliferation was analyzed following the Cell Count Kit-8 (Dojindo Laboratories, Kumamoto, Japan) operating manual. A microplate reader, supplied by Thermo Fisher Scientific, Waltham, MA, USA, was adopted to read the absorbance_450nm_.

### 2.7. Flow Cytometry Assay

90% confluent cells were washed with PBS for 2 to 3 times. Then, cell digestion with trypsin-EDTA solution and resuspension in 500 *μ*L binding buffer were performed. Subsequently, the cell resuspension was stained with a mixture comprising allophycocyanin (APC) and phycoerythrin (PE), both supplied by Sigma-Aldrich with an amount of 5 *μ*L, for 15 min at an ambient temperature in a dark environment. Flow cytometry (BD FACSVerse, USA) determined the apoptosis rate.

### 2.8. Immunofluorescence Assay

Cells were maintained and adhered on chamber slides. After triple PBS rinses, they were treated with 4% paraformaldehyde fixation (10 min), 1% BSA blocking, and overnight cultivation (4°C) with the Iba1 antibody (1 : 1000, ab48004, Abcam). Subsequently, they were processed for triple PBS washes and 60 min of goat anti-rat IgG H&L (Alexa Fluor® 647) (1 : 500, ab150167, Abcam) incubation (37°C). This was followed by nuclear staining with DAPI (C1002, Beyotime, Shanghai, China), and the final image was captured with a confocal microscopy (LSM700; Zeiss, Oberkochen, Germany).

The article "CX3CL1 Derived from Bone Marrow Mesenchymal Stem Cells Inhibits Aβ1-42-Induced SH-SY5Y Cell Pathological Damage through TXNIP/NLRP3 Signaling Pathway" was retracted in 2023. Reasons: unreliable results or conclusions; concerns about the data; concerns about the peer review; concerns about the citations.

### 2.9. MDA, SOD, CAT, and GSH-Px Measurements

Malondialdehyde (MDA), superoxide dismutase (SOD), catalase (CAT), and glutathione peroxidase (GSH-Px) measurements used MDA (A003-1-1), total SOD (T-SOD) (A001-1-1), CAT (A007-1-1), and GSH-Px test kits (A005-1-2; all from Nanjing Jiancheng Bioengineering Institute, China), respectively, following the operating manual of the corresponding kit. The microplate reader read the absorbance of wells at 532, 560, 405, and 412 nm for MDA, SOD, CAT, and GSH, respectively.

### 2.10. Statistical Processing

All data collected were present in the form of the mean ± standard deviation, and the statistical significance threshold was *p* < 0.05. Each assay was replicated 3 times. One-way analysis of variance and Duncan's test were employed to identify inter- and multigroup differences, respectively. SPSS 20.0 (SPSS Inc., Chicago, IL, USA) was used for analysis.

## 3. Results

### 3.1. BMSC-Derived CX3CL1 Reversed the A*β*_1-42_-Reduced Level of CX3CL1 in SH-SY5Y

To explore the role played by CX3CL1 derived from BMSCs in a A*β*_1-42_-induced SH-SY5Y cell model, pcDNA-ligated CX3CL1 overexpression plasmid was first transfected into BMSCs to upregulate CX3CL1 expression in BMSCs. ELISA (Figure 1(a)) and western blotting (Figures 1(b) and 1(c)) results showed that overexpression of CX3CL1 in BMSCs observably increased the levels of both soluble and membrane-bound CX3CL1, while there were no differences between the NC-ov and control groups. Besides, statistically decreased soluble and membrane-bound CX3CL1 levels were observed in SH-SY5Y under A*β*_1-42_ inducement, which were significantly rescued by the coculture of BMSCs (Figures 1(d)–1(f)). Moreover, overexpression of CX3CL1 in BMSCs further statistically enhanced CX3CL1 levels of both the soluble and membrane-bound forms, whereas transfection of NC-ov showed no statistical effect (Figures 1(d)–1(f)). These results indicated that CX3CL1 derived from BMSCs notably reversed the A*β*_1-42_-reduced CX3CL1 expression in SH-SY5Y cells.

### 3.2. CX3CL1 Derived from BMSCs Increased A*β*_1-42_-Induced SH-SY5Y Viability but Suppressed Apoptosis

Then, we investigated the role played by CX3CL1 derived from BMSCs in SH-SY5Y cell growth under A*β*_1-42_ inducement. Statistically declined A*β*_1-42_-intervened SH-SY5Y cell viability was found compared to the control group, which was markedly inverted by the coculture of BMSCs (Figure 2(a)). Also, transfection of CX3CL1 overexpression plasmid (not empty plasmid) into BMSCs further markedly elevated SH-SY5Y cell viability compared to SH-SY5Y with A*β*_1-42_ and BMSC coculture (Figure 2(a)). However, the opposite tendency was discovered in SH-SY5Y cell apoptosis, as indicated by that cocultured with BMSCs significantly reduced the A*β*_1-42_-increased apoptosis rate (Figures 2(b) and 2(c)) and the relative protein expression of cleaved caspase-3 (Figures 2(d) and 2(e)) of SH-SY5Y cells, which was prominently antagonized with the overexpression of CX3CL1 in BMSCs. These data suggested that CX3CL1 derived from BMSCs significantly enhanced A*β*_1-42_-induced SH-SY5Y cell growth but inhibited apoptosis.

The article "CX3CL1 Derived from Bone Marrow Mesenchymal Stem Cells Inhibits Aβ1-42-Induced SH-SY5Y Cell Pathological Damage through TXNIP/NLRP3 Signaling Pathway" was retracted in 2023. Reasons: unreliable results or conclusions; concerns about the data; concerns about the peer review; concerns about the citations.

### 3.3. CX3CL1 Derived from BMSCs Ameliorated the Pathology-Induced A*β*_1-42_ in SH-SY5Y

Next, the role played by CX3CL1 derived from BMSCs in the pathology of A*β*_1-42_-induced SH-SY5Y was investigated. A*β*, tau, and p-Tau were found to be markedly increased with the induction of A*β*_1-42_ in SH-SY5Y, which was statistically improved with the coculture of BMSCs (Figures 3(a)–3(d)). Moreover, transfection of CX3CL1 overexpression plasmid (not empty plasmid) into BMSCs further notably diminished the relative protein expression of A*β*, tau, and p-Tau (Figures 3(a)–3(d)). Also, similar changes were found in the relative integrated density of Iba1 (Figures 3(e) and 3(f)). Besides, coculture of BMSCs obviously improved the cell growth and axon length of A*β*_1-42_-induced SH-SY5Y, which was further ameliorated with the overexpression of CX3CL1 in BMSCs (Figure 3(g)). Furthermore, the relative protein expressions of synaptic markers, including SNAP25, Synapsin1, and PSD95, were statistically declined in SH-SY5Y with A*β*_1-42_ inducement, which were notably reversed by the coculture of BMSCs (Figures 3(h)–3(k)). Consistently, upregulation of CX3CL1 in BMSCs further statistically elevated SNAP25, Synapsin1, and PSD95 protein levels (Figures 3(h)–3(k)). Taken together, these results demonstrated that CX3CL1 derived from BMSCs obviously improved the pathology-induced A*β*_1-42_ in SH-SY5Y.

### 3.4. The Influence of BMSC-Derived CX3CL1 on A*β*_1-42_-Induced SH-SY5Y Was Associated with TXNIP/NLRP3 Axis

Furthermore, the potential mechanisms associated with the role of CX3CL1 derived from BMSCs in SH-SY5Y with A*β*_1-42_ inducement were studied. Coculture of BMSCs markedly declined the A*β*_1-42_-enhanced MDA concentration, which was further statistically decreased by overexpression of CX3CL1 in BMSCs (Figure 4(a)). On the contrary, coculture of BMSCs markedly elevated the A*β*_1-42_-reduced concentrations of SOD, CAT, and GSH-Px, which was further significantly increased by overexpression of CX3CL1 in BMSCs (Figures 4(b)–4(d)). Mechanically, coculture of BMSCs prominently diminished the A*β*_1-42_-enhanced TXNIP and NLRP3 protein levels while aggrandized the A*β*_1-42_-attenuated Trx protein expression (Figures 4(e)–4(h)). Moreover, upregulation of CX3CL1 in BMSCs further statistically strengthened the corresponding tendency (Figures 4(e)–4(h)). Together, these data clarified that the effect of CX3CL1 derived from BMSCs on A*β*_1-42_-induced SH-SY5Y involved the TXNIP/NLRP3 signaling axis.

The article "CX3CL1 Derived from Bone Marrow Mesenchymal Stem Cells Inhibits Aβ1-42-Induced SH-SY5Y Cell Pathological Damage through TXNIP/NLRP3 Signaling Pathway" was retracted in 2023. Reasons: unreliable results or conclusions; concerns about the data; concerns about the peer review; concerns about the citations.

## 4. Discussion

AD is the most prevalent neurodegenerative brain disorder that imposes a severe burden on patients and their families, even leading to social and economic losses [30]. It is demonstrated that MSC therapy is a novel and promising treatment for AD, whose paracrine action is meant to trigger immunomodulation and neural regeneration [17]. CX3CL1 is essential in the regulation of microglia activation, neuroprotection, and immunomodulation by MSCs [20, 21]. In this paper, A*β*_1-42_ treatment markedly reduced both soluble and membrane-bound CX3CL1 levels, cell viability, protein levels of synaptic markers (SNAP25, Synapsin1, and PSD95), SOD, CAT, and GSH-Px concentrations, and Trx protein expression, while it enhanced apoptosis, cleaved caspase-3, A*β*, tau, and p-Tau protein levels, relative integrated density of Iba1, MDA concentration, and TXNIP and NLRP3 protein levels in SH-SY5Y; however, the above effects were prominently reversed by the coculture of BMSCs. Moreover, we overexpressed CX3CL1 in BMSCs and found that overexpression of CX3CL1 in BMSCs observably strengthened the corresponding tendency caused by the coculture of BMSCs.

The membrane-bound CX3CL1 and soluble CX3CL1 play diverse roles under physiological conditions. Membrane-bound CX3CL1 functions is involved in infiltrating leukocyte recruitment and adhesion [31], while soluble CX3CL1 serves as a chemoattractant associated with the cellular migration, as well as a neuroprotective signaling molecule to contribute to the sustainability of the resting state of microglia [32, 33]. Besides, soluble CX3CL1 modulates the anti-inflammatory effect in the brain, and the receptors of membrane-bound CX3CL1 are located on microglial cell surfaces [32, 34]. During fibrosis amelioration, MSCs can participate in Ly-6C-high (inflammatory) to Ly-6C low (anti-inflammatory) macrophage polarization by increasing CX3CL1 levels, exerting significant effects on ameliorating liver disease [35]. The cerebrospinal fluid CX3CL1 level is reported to be notably diminished in AD patients [36]. Also, our results revealed statistically reduced soluble and membrane-bound CX3CL1 levels in SH-SY5Y cells under A*β*_1-42_ inducement. However, coculture of BMSCs markedly rescued decreased CX3CL1 by A*β*_1-42_ in SH-SY5Y, implying that BMSCs might express and secrete CX3CL1 to compensate for the loss of CX3CL1 [37]. Overexpression of CX3CL1 in BMSCs further confirmed this conclusion. Besides, we discovered that CX3CL1 derived from BMSCs significantly enhanced A*β*_1-42_-induced SH-SY5Y growth but declined apoptosis rate and cleaved caspase-3 at the protein level. Cleaved caspase-3 is the activation form of caspase-3 that can regulate different phases of the apoptotic pathway [38]. Therefore, these findings elucidated that A*β*_1-42_ treatment resulted in low level of CX3CL1, which was positively associated with the growth and negatively related to the apoptosis of SH-SY5Y cells. Upregulation of CX3CL1 in BMSCs obviously increased the reduced CX3CL1 and proliferation of SH-SY5Y cells but inhibited increased apoptosis by A*β*_1-42_. Taken together, CX3CL1 derived from BMSCs reversed the A*β*_1-42_-reduced CX3CL1, which increased the viability but suppressed the apoptosis of SH-SY5Y under A*β*_1-42_ inducement.

The article "CX3CL1 Derived from Bone Marrow Mesenchymal Stem Cells Inhibits Aβ1-42-Induced SH-SY5Y Cell Pathological Damage through TXNIP/NLRP3 Signaling Pathway" was retracted in 2023. Reasons: unreliable results or conclusions; concerns about the data; concerns about the peer review; concerns about the citations.

A*β* accumulation and hyperphosphorylated tau are the dominating pathological hallmarks of AD [39, 40], which may explain prominently high A*β*, Tau, and p-Tau protein levels in SH-SY5Y with A*β*_1-42_ inducement in this research. Recently, Qin et al. [41] have reported that BMSC transplantation mitigated neuropathology and ameliorated cognitive deficits in AD animal models. Consistently, we found that coculture of BMSCs statistically reduced the A*β*_1-42_-increased A*β*, Tau, and p-Tau protein levels, which were further notably decreased by the upregulation of CX3CL1 in BMSCs. Tau and A*β* are the prime suspects driving AD pathology and, as such, have become the focus of therapeutic development. There is mounting evidence that these proteins may perform many crucial physiological functions during AD pathological development that can be disrupted by A*β*- or tau-lowering therapeutics [42]. In the past decades, a large number of research has demonstrated that neuroinflammation is a central risk factor of AD; thus, strategies of decreasing neuroinflammation have been regarded as the promising therapeutics for AD [43, 44]. Neuroinflammation in the brain is mediated by microglial cells, so microglial activation is a characteristic of neuroinflammation [45, 46]. Here, we observed that coculture of BMSCs significantly declined the A*β*_1-42_-enhanced relative integrated density of Iba1, a marker of microglial cells, which was further obviously diminished by the overexpression of CX3CL1 in BMSCs, indicating that CX3CL1 derived from BMSCs inhibited neuroinflammation in SH-SY5Y with A*β*_1-42_ inducement. Moreover, it confirmed the fact that soluble CX3CL1 plays an anti-inflammatory role in the brain [32, 34]. In addition, it has been demonstrated that A*β* and Tau oligomers, as well as neuroinflammation, can conduce to synaptic loss, which results in synaptic dysfunction [46–48]. Our findings revealed that coculture of BMSCs obviously improved A*β*_1-42_-induced SH-SY5Y cell growth and axon length, which was further notably ameliorated by the overexpression of CX3CL1 in BMSCs. Also, coculture of BMSCs statistically elevated the A*β*_1-42_-attenuated relative protein levels of SNAP25, Synapsin1, and PSD95, as well as the presynaptic and postsynaptic markers, which was further markedly promoted by the overexpression of CX3CL1 in BMSCs. Based on the above, we can draw the conclusion that CX3CL1 derived from BMSCs notably suppressed pathological damage in A*β*_1-42_-induced SH-SY5Y cells.

The article "CX3CL1 Derived from Bone Marrow Mesenchymal Stem Cells Inhibits Aβ1-42-Induced SH-SY5Y Cell Pathological Damage through TXNIP/NLRP3 Signaling Pathway" was retracted in 2023. Reasons: unreliable results or conclusions; concerns about the data; concerns about the peer review; concerns about the citations.

Furthermore, neuroinflammation can induce oxidative stress in the brain [48]. In the present study, A*β*_1-42_ treatment remarkably reduced SOD, CAT, and GSH-Px concentrations in SH-SY5Y while enhancing MDA levels, which were prominently reversed by the coculture of BMSCs. Overexpression of CX3CL1 in BMSCs observably strengthened the corresponding tendency caused by the coculture of BMSCs, which suggested statistically inhibited oxidative stress in SH-SY5Y with A*β*_1-42_ inducement by BMSC-derived CX3CL1. TrX is an intracellular antioxidative protein via thiol reduction and the scavenging of reactive oxygen species (ROS) [49]. This research identified that TrX expression was predominately decreased in SH-SY5Y with A*β*_1-42_ inducement, which was in line with the reduction in AD brain regions [50]. TrX can be bound by TXNIP to dampen TrX activation and facilitate oxidative stress [51]. Oakley et al. [52] exhibited that the level of TXNIP was upregulated in the hippocampus of mice in a 5 × AD mouse model. Consistently, SH-SY5Y with A*β*_1-42_ inducement presented overexpressed TXNIP in our study. Moreover, TXNIP is a key link between inflammasome activation and oxidative stress [53]. Under oxidative stress, dissociated TXNIP from TrX binds to NLRP3 that conduces to inflammasome formation and activation. Consequently, a series of proinflammatory mediators are secreted to enhance neuroinflammation, which promotes synaptic dysfunction and the subsequent AD progression. Furthermore, Wang et al. [54] have reported an enhancement of binding between TXNIP and NLRP3 in the APP/PS1 mouse brain, and NLRP3 inflammasome and Nrf2/TXNIP/TrX axis are involved in the pathological changes of AD. Here, we discovered that A*β*_1-42_ treatment notably decreased Trx protein expression and elevated TXNIP and NLRP3 protein levels in SH-SY5Y that were prominently reversed by the coculture of BMSCs. Upregulation of CX3CL1 in BMSCs significantly intensified the corresponding tendency caused by the coculture of BMSCs. Therefore, these results elaborated that the role of CX3CL1 derived from BMSCs in A*β*_1-42_-iintervened SH-SY5Y was linked to the TXNIP/NLRP3 signaling axis.

The article "CX3CL1 Derived from Bone Marrow Mesenchymal Stem Cells Inhibits Aβ1-42-Induced SH-SY5Y Cell Pathological Damage through TXNIP/NLRP3 Signaling Pathway" was retracted in 2023. Reasons: unreliable results or conclusions; concerns about the data; concerns about the peer review; concerns about the citations.

## 5. Conclusion

In conclusion, our results revealed that through the TXNIP/NLRP3 signaling pathway, CX3CL1 derived from BMSCs alleviates A*β*_1-42_-induced SH-SY5Y cell injury. However, there are still some limitations in our study. First, Lee et al. [55] have reported that membrane-bound CX3CL1 but not soluble CX3CL1 mediated the A*β* pathology. Our results showed that CX3CL1 derived from BMSCs reversed the A*β*_1-42_-reduced soluble and membrane-bound CX3CL1 levels; hence, whether the membrane-bound CX3CL1 consistently improved the A*β* pathology or not needs further exploration in our subsequent studies. Besides, multiple research has demonstrated that the CX3CL1 is closely involved in inflammation [56–58]. However, in our study, we failed to further reveal the role of CX3CL1 derived from BMSCs in neuroinflammation. Also, the findings are not verified in vivo. Thus, more experiments are expected to be conducted in further studies to explore the underlying mechanism. In brief, it is hoped that our results can lay a foundation for AD treatment and even the management of other neurodegenerative disorders.

## Figures and Tables

**Figure 1:** CX3CL1 derived from BMSCs significantly inverted A*β*_1-42_-decreased CX3CL1 in SH-SY5Y. (a) Soluble CX3CL1 expression in BMSCs was detected by ELISA. (b and c) Western blotting determined CX3CL1 expression relative to *β*-actin in BMSCs. (d) ELISA measured soluble CX3CL1 levels in SH-SY5Y under different interventions. (e and f) Western blotting examined CX3CL1 expression relative to *β*-actin in SH-SY5Y under different interventions. ns: nonsignificance; ^∗^*p* < 0.05 versus control group; ^#^*p* < 0.05 versus A*β* group; ^&^*p* < 0.05 versus A*β*+MSC group.

**Figure 2:** CX3CL1 derived from BMSCs statistically augmented A*β*_1-42_-induced SH-SY5Y viability but repressed apoptosis. (a) CCK-8 assay assessed SH-SY5Y viability. (b and c) Flow cytometry evaluated SH-SY5Y apoptosis. (d and e) Western blotting determined cleaved caspase-3 expression relative to *β*-actin. ^∗^*p* < 0.05 versus control group; ^#^*p* < 0.05 versus A*β* group; ^&^*p* < 0.05 versus A*β*+MSC group.

**Figure 3:** CX3CL1 derived from BMSCs alleviated the pathology-induced A*β*_1-42_ in SH-SY5Y. (a–d) Western blotting examined A*β*, tau, and p-Tau protein expressions relative to *β*-actin. (e and f) The relative integrated density of Iba1 was evaluated by IF. (g) The axons of SH-SY5Y cells were observed using inverted microscope. (h–k) Western blotting examined SNAP25, Synapsin1, and PSD95 protein levels relative to *β*-actin. ^∗^*p* < 0.05 versus control group; ^#^*p* < 0.05 versus A*β* group; ^&^*p* < 0.05 versus A*β*+MSC group.

The article "CX3CL1 Derived from Bone Marrow Mesenchymal Stem Cells Inhibits Aβ1-42-Induced SH-SY5Y Cell Pathological Damage through TXNIP/NLRP3 Signaling Pathway" was retracted in 2023. Reasons: unreliable results or conclusions; concerns about the data; concerns about the peer review; concerns about the citations.

**Figure 4:** The role played by CX3CL1 derived from BMSCs in A*β*_1-42_-induced SH-SY5Y was related to TXNIP/NLRP3 axis. (a–d) MDA, SOD, CAT, and GSH-Px concentrations measured by commercial kits. (e–h) Western blotting tested TXNIP, NLRP3, and Trx protein levels relative to *β*-actin. ^∗^*p* < 0.05 versus control group; ^#^*p* < 0.05 versus A*β* group; ^&^*p* < 0.05 versus A*β*+MSC group.

## Data Availability

The data sets used and analyzed during the current study are available from the corresponding author on reasonable request.
